The article "Mathematical Modeling and Control of COVID-19 Using Super Twisting Sliding Mode and Nonlinear Techniques" was published in 2022. Journal: Comput Intell Neurosci.

# Mathematical Modeling and Control of COVID-19 Using Super Twisting Sliding Mode and Nonlinear Techniques

**DOI:** 10.1155/2022/8539278

**Published:** 2022-06-30

**Authors:** Anwer S. Aljuboury, Firas Abedi, Hanan M. Shukur, Zahraa Sabah Hashim, Ibraheem Kasim Ibraheem, Ahmed Alkhayyat

**Affiliations:** ^1^Continuing Education Center, Mustansiriyah University, Baghdad 14022, Iraq; ^2^Information Technology Unit, Hilla University College, Babylon 51001, Iraq; ^3^Department of Mathematics, College of Education, Al-zahraa University for Women, Karbala, Iraq; ^4^Computer Techniques Engineering Dept., Al-Kitab University, Kirkuk, Iraq; ^5^Department of Electrical Engineering, College of Engineering, University of Baghdad, Baghdad 10001, Iraq; ^6^Department of Computer Techniques Engineering, Dijlah University College, Baghdad 10001, Iraq; ^7^College of Technical Engineering, the Islamic University, Najaf, Iraq

## Abstract

Since the outbreak of the COVID-19 epidemic, several control strategies have been proposed. The rapid spread of COVID-19 globally, allied with the fact that COVID-19 is a serious threat to people's health and life, motivated many researchers around the world to investigate new methods and techniques to control its spread and offer treatment. Currently, the most effective approach to containing SARS-CoV-2 (COVID-19) and minimizing its impact on education and the economy remains a vaccination control strategy, however. In this paper, a modified version of the susceptible, exposed, infectious, and recovered (SEIR) model using vaccination control with a novel construct of active disturbance rejection control (ADRC) is thus used to generate a proper vaccination control scheme by rejecting those disturbances that might possibly affect the system. For the COVID-19 system, which has a unit relative degree, a new structure for the ADRC has been introduced by embedding the tracking differentiator (TD) in the control unit to obtain an error signal and its derivative. Two further novel nonlinear controllers, the nonlinear PID and a super twisting sliding mode (STC-SM) were also used with the TD to develop a new version of the nonlinear state error feedback (NLSEF), while a new nonlinear extended state observer (NLESO) was introduced to estimate the system state and total disturbance. The final simulation results show that the proposed methods achieve excellent performance compared to conventional active disturbance rejection controls.

## 1. Introduction

COVID-19 has become one of the most dangerous pandemics in recent global history, with over 198 million confirmed cases and 4.237 million deaths as of 1 August 2021, according to the World Health Organization (WHO) [1]. Various control strategies have thus been proposed and tested to suppress or even reduce the spread of SARS-CoV-2.

Various authors [2–7] have presented mathematical models and the analyses of COVID-19, while others [8–12] have sought to use optimal control theory to stem the COVID-19 pandemic via measures such as social distancing, quarantine, contact tracing, case detection, imposition of face masks, media coverage, and other suppression and mitigation strategies. In [13], a firm control technique was used with a variable transformation technique (VTT) and most valuable player algorithm (MVPA) as a way to control the unstable behavior of a COVID-19 nonlinear model to reduce spread, while in [14, 15], a PID controller was used to stem the rapid spread of the COVID-19 pandemic. However, the aforementioned studies did not take into account the effect of disturbance or uncertainty into consideration. The authors of [16] introduced the extended state observer with a U-model control-based city lockdown strategy with the population size that is unknown, which can be considered as a disturbance to show the effectiveness of the proposed method, and [17] used various nonlinear models of COVID-19 alongside various control strategies such as vaccination, shielding and immunity, and quarantine by applying a metric temporal logic (MTL) formula. The author in [18] introduced a new control technique to remove disturbances and parameter uncertainty effects within linear or nonlinear systems, while the authors in [19–22] presented the design and analysis of a super twisting sliding mode controller (STC-SM) with respect to various systems, including three-phase grid-connected photovoltaic, pneumatic muscle actuators, aircraft at a high angle of attack, and microgyroscopes. In addition to that, a review of different schemes of the sliding mode controller for the network system is introduced in [23]. A nonlinear extended state observer (NLESO) was also introduced in [24, 25].

Although various control strategies have been proposed to address the COVID-19 pandemic, many of these suffer from severe drawbacks: for example, most of them treat the control signal as a constant or take insufficient account of disturbances that may increase the spread COVID-19, such as bad weather, failure to commit to health measures, and failure to distribute vaccinations in a fair manner between countries, especially the poor ones. The exception is [16], which takes uncertainty around population numbers as a source of the disturbance. However, none of the listed studies has applied a vaccination control strategy with robust control and ADRC techniques.

Motivated by this gap, this paper presents the proposed nonlinear model of COVID-19, utilizing a vaccination control strategy that takes account of the noted exogenous disturbances. Furthermore, a novel nonlinear controller with an unprecedented tracking differentiator and a new nonlinear extended state observer were applied, generating the combination necessary to support a new proposed ADRC for the COVID-19 nonlinear system with a rapid output response with noise reduction due to the use of TD with the proposed nonlinear PID (NLPID) controller and the proposed super twisting sliding mode (STC-SM) controller. The parameters of the proposed nonlinear PID (NLPID) controller, proposed super twisting sliding mode (STC-SM) controller, proposed nonlinear ESO (NLESO), and tracking differentiator are tuned using a genetic algorithm, and a multiobjective performance index is used in the minimization process, which includes the absolute values of the control signals and the square of the control signals.

The rest of this paper is organized as follows: Section 2 presents the modeling of the COVID-19 system, and Section 3 presents the proposed ADRC.  Section 4 introduces the convergence of the NLESO and the idea of closed-loop stability, allowing the simulation results and *q* discussion of the results to be demonstrated in Section 5. Finally, the conclusion of this paper is presented in Section 6.

## 2. COVID-19 Mathematical Model

The proposed nonlinear mathematical model of the COVID-19 system is developed from the model in [17]. In this model, the population is divided into seven classes: the susceptible, the exposed, the infected, the hospitalized infected, the cumulative infected, the dead, and the recovered. As shown in the flow diagram in Figure 1, the proposed nonlinear model of the COVID-19 with vaccination strategy is thus as follows:

(1) $$\begin{array}{c} \dot{I}=\epsilon_{\text{COV}}E-\left(\gamma_{\text{COV}}+\mu_{\text{COV}}+\alpha_{\text{COV}}+b_{\text{COV}}\right)I, \end{array}$$

(2) $$\begin{array}{c} \dot{E}=\frac{\beta_{\text{COV}}\text{IS}}{N_{\text{COV}}}-\left(\mu_{\text{COV}}+\epsilon_{\text{COV}}\right)E, \end{array}$$

(3) $$\begin{array}{c} \dot{S}=\lambda_{\text{COV}}N_{\text{COV}}-\mu_{\text{COV}}S-\frac{\beta_{\text{COV}}\text{IS}}{N_{\text{COV}}}-V, \end{array}$$

(4) $$\begin{array}{c} \dot{H}=b_{\text{COV}}I-\left(\gamma_{\text{COV}}+\mu_{\text{COV}}\right)H, \end{array}$$

(5) $$\begin{array}{c} \dot{C}=b_{\text{COV}}I, \end{array}$$

(6) $$\begin{array}{c} \dot{R}=\gamma_{\text{COV}}I-\mu_{\text{COV}}R+\left(V+\text{d}\right), \end{array}$$

(7) $$\begin{array}{c} \dot{D}=\alpha_{\text{COV}}I+\alpha_{\text{COV}}H, \end{array}$$

where *V* is the number of vaccinated people per day (the controlled input), and *S*, *E*, *I*, *H*, *C*, and *R* denote the susceptible, exposed, infected, hospitalized infected, cumulative infected, and recovered populations, respectively. Additionally, in this model, *N*_COV_ > 0 is the total population,; *D* represents the number of deaths caused by COVID-19, and *ϵ*_COV_, *μ*_COV_, *α*_COV_, *b*_COV_, *γ*_COV_, *β*_COV_,  and *λ*_COV_ are the rates of progression from *E* to *I* (the reciprocal of the incubation period), the per capita natural death rate, the SARS-CoV-2 virus-induced average fatality, the diagnosis rate, the recovery rate of infectious individuals, the probability of disease transmission per contact (transmission rate), and the per capita birth rate, respectively. The value *d* is the exogenous disturbance of the system. All parameters are assumed to be positive, and where the birth rate is equal to the death rate (*μ*_COV_=*λ*_COV_), the total population size may be considered constant over time. Thus, $\dot{N}\left(t\right)=\dot{S}+\dot{E}+\dot{I}+\dot{H}+\dot{R}$ illustrates the dynamics of total population size ${\dot{N}}_{\text{COV}}=0$.

## 3. Active Disturbance Rejection Control Design

The active disturbance rejection control (ADRC) was first proposed by [18], and it is now considered one of the most accurate and powerful control techniques for estimating the unwanted disturbances, system dynamics, and parameter variation often denoted as “generalized disturbances.” The ADRC segments work in a complementary manner whereby the tracking differentiator (TD) offers a smooth reference with its derivate and the nonlinear state error feedback (NLSEF) draws the required information for the plant from the extended state observer (ESO), in order to control the system; meanwhile, the ESO estimates the internal and external disturbance and actively cancels it. The ADRC is thus suitable for systems with a relative degree of two or higher.  Figure 2 shows the general form of the ADRC.

In this paper, the ADRC for a system with a relative degree of one is introduced by combining the proposed tracking differentiator with the NLSEF to form a new control frame for the ADRC. The general form of the proposed unit relative degree ADRC is shown in Figure 3: this consists of three parts described in more detail below.

### 3.1. Proposed Tracking Differentiator (TD)

In order to generate an accurate and smooth differentiated signal from the reference signal, avoiding set point jumping and achieving fast tracking, a TD is utilized. This TD limits the high-frequency oscillations, allowing the differentiated output signal to become more sensitive to noise. As mentioned previously, the tracking differentiator is generally second-order or higher; however, for *ρ*=1, using the TD has previously been avoided because the extended state observer estimates two states (i.e., *z*_1_ and *z*_2_). For the purposes of this paper, however, it is possible to use the tracking differentiator in a unit relative degree system, utilizing the mathematical representation of TD for *ρ*=1 given as

(8) $$\begin{array}{c} \left\{\begin{array}{c} {\dot{\tilde{e}}}_{1}={\tilde{e}}_{2},\\ {\dot{\tilde{e}}}_{2}=-a_{1}R^{2}\left(\frac{{\tilde{e}}_{1}-\tilde{e}}{\sqrt{1+{\left({\tilde{e}}_{1}-\tilde{e}\right)}^{2}}}\right)-a_{2}R{\tilde{e}}_{2}, \end{array}\right) \end{array}$$

(9) $$\begin{array}{c} \left\{\begin{array}{c} {\dot{\tilde{e}}}_{1}={\tilde{e}}_{2},\\ {\dot{\tilde{e}}}_{2}=-a_{1}R^{2}\left(\frac{{\tilde{e}}_{1}-\tilde{e}}{1+\left|{\tilde{e}}_{1}-\tilde{e}\right|}\right)-a_{2}R{\tilde{e}}_{2}, \end{array}\right) \end{array}$$

where ${\tilde{e}}_{1}$ and ${\tilde{e}}_{2}$ are the tracking error and the tracking error derivative, respectively, and $\tilde{e}$ is the input error to the TD. Thus, *R* is a positive tuning parameter that is chosen depending on the application, and *a*_1_ and *a*_2_ are tuning parameters. As shown in equations (8) and (9), the error becomes the input to the tracking differentiator rather than the reference signal, and the result is a smooth original signal and its derivative that avoids chatter in the output signal. In the proposed TD, the sigmoid function (2) and Elliott squash function (equation (9) given in [26] are utilized instead of the sign function used in the conventional tracking differentiator proposed by [18], however.

### 3.2. Proposed Controller

In this paper, two nonlinear controllers are proposed as NLSEF, which can be further defined as follows.

#### 3.2.1. NLPID-TD

The NLPID controller is the developed version of the LPID; this is necessary to handle the strong nonlinearity of the COVID-19 system, which cannot be addressed using the linear version. The proposed NLPID thus depends on nonlinear functions, particularly the sign function and exponential function. The proposed NLPID can thus be given as

(10) $$\begin{array}{c} \left\{\begin{array}{c} u_{1}=\frac{k_{1}}{1+\text{exp}\left({\tilde{e}}_{1}^{2}\right)}{\left|{\tilde{e}}_{1}\right|}^{\alpha_{1}}\text{sign}\left({\tilde{e}}_{1}\right),\\ u_{2}=\frac{k_{2}}{1+\text{exp}\left({\dot{\tilde{e}}}_{1}^{2}\right)}{\left|{\dot{\tilde{e}}}_{1}\right|}^{\alpha_{2}}\text{sign}\left({\dot{\tilde{e}}}_{1}\right),\\ u_{3}=\frac{k}{1+\text{exp}\left(\int {\tilde{e}}_{1}^{2}\right)}{\left|{\tilde{e}}_{1}\right|}^{\alpha_{3}}\text{sign}\left(\int {\tilde{e}}_{1}\text{d}t\right),\\ u_{0_{\text{NLPD}}}=u_{1}+u_{2}+u_{3}, \end{array}\right) \end{array}$$

where *k*_1_, *k*_2_, *k*_3_, *α*_1_, *α*_2_ and *α*_3_ are tuning design parameters and ${\dot{\tilde{e}}}_{1}={\tilde{e}}_{2}$. Moreover, *α*_1_, *α*_2_, and*α*_3_ < 1 to ensure that the error functions ${\left|\tilde{e}\right|}^{\alpha_{1}}$, ${\left|{\tilde{e}}_{1}\right|}^{\alpha_{2}},\text{ and}{\left|{\dot{\tilde{e}}}_{1}\right|}^{\alpha_{3}}$ are sensitive to small error values. The combination of the proposed NLPID controller and the proposed tracking differentiator showed excellent results in terms of controlling the spread of COVID-19.

#### 3.2.2. Proposed Super Twisting Sliding Mode Controller (STC-SM)

To avoid the problem of chatter, a conventional super twisting controller (CST-SMC) is utilized. This offers a second-order sliding mode in the nonlinear version of the PI controller, which is designed for a system with a relative degree of one [19, 26]. The STC-SM guarantees that trajectories can reach the sliding surface and converge in a finite amount of time because the trajectories twist around the origin of the sliding surface; the STC-SM thus guarantees this continuity and convergence in finite time by replacing the term *b*∫sign(*σ*) with a continuous function, which has several advantages. One of these advantages is the shape of the signal, which is S-shaped and produces a more rapid rise in the value of the result; in addition, the range is bounded between [*x*, −*x*], which saturates the value without creating a sharp edge. The proposed STC-SM can thus be expressed as follows:

(11) $$\begin{array}{c} \varsigma =\kappa {\tilde{e}}_{1}+{\dot{\tilde{e}}}_{1}, \end{array}$$

(12) $$\begin{array}{c} u_{0_{\text{STC}-\text{SM}}}=\kappa {\left|\varsigma \right|}^{p}\text{sign}\left(\varsigma \right)+\xi \text{tan}h\left(\frac{\varsigma }{\delta }\right), \end{array}$$

where *ς* is the sliding surface; *κ* is sliding coefficient and a positive tuning parameter; ${\tilde{e}}_{1}$ and ${\dot{\tilde{e}}}_{1}$ are the tracking error and its derivative, respectively; *ξ*  is sliding coefficient; and *p* and *δ*  are positive values that need to be tuned to achieve the optimal value parameters, such that 0 < *p* < 1 and *δ* > 0. It is important to note that *ς* is selected in such ways that guarantee that the equation (i.e., equation (11)) is stable. Thus, as can be seen from equation (11), the sliding surface is selected that depends on the error and its derivative obtained from the tracking differentiator mentioned previously and the sliding coefficient that is considered a tuning parameter in this paper.

### 3.3. Proposed Nonlinear Extended State Observer (NLESO)

In order to solve the problem of peaking that may appear in a linear ESO, a nonlinear extended state observer (NLESO) is utilized. The proposed NLESO is designed to estimate external disturbances, internal dynamics, and uncertainty, expressed as follows:

(13) $$\begin{array}{c} \left\{\begin{array}{c} {\dot{z}}_{1}=z_{2}+b_{0}u+\beta_{1}{\hat{e}}_{1},\\ {\dot{z}}_{2}=\beta_{2}{\hat{e}}_{2}, \end{array}\right) \end{array}$$

(14) $$\begin{array}{c} \left\{\begin{array}{c} {\hat{e}}_{1}=\text{sign}\left(e_{1}\right){\left|e_{1}\right|}^{p_{1}}+Ae_{1},\\ {\hat{e}}_{2}=\text{sign}\left(e_{1}\right){\left|e_{1}\right|}^{p_{1}/2}+Ae_{1}, \end{array}\right) \end{array}$$

where *e*_1_ = *S* − *z*_1_, *e*_1_ is the estimation error, *z*_1_ is the estimation state of *S*, ${\hat{e}}_{1}$ and ${\hat{e}}_{2}$ are the nonlinear functions, *p*_1_ is a tuning parameter of less than 1, *𝒜* is a tuning parameter, and *β*_1_ and *β*_2_ are the observer gain parameters, selected in such a way that the characteristic polynomial *s*^2^+*β*_1_*s*+*β*_2_=(*ω*_0_+*s*)^2^ is Hurwitz [27, 28]. Thus, *ω*_0_ is the NLESO bandwidth, and *b*_0_ is the approximated parameter of *b* in the system. The proposed ADRC with a nonlinear model of the COVID-19 system is thus shown in Figure 4.

## 4. Closed-Loop Stability Analysis

The convergence of the proposed NLESO and the closed-loop stability of the overall system are introduced in this section and stated in the sequence below.

### 4.1. The Convergence of the Proposed NLESO

In this subsection, the convergence of the proposed NLESO is analyzed and demonstrated using the Lyapunov stability criterion.

The error dynamics can be written as follows: equations (1)–(7) can be rewritten in Brunovesky form:

Let *x*_1_=*S*, $x_{2}=\dot{S}$, and *x*=[*I* *E* *H* *C* *R*  *D*], then

(15) $$\begin{array}{c} \left\{\begin{array}{c} {\dot{x}}_{1}=x_{2},\\ {\dot{x}}_{2}=Ϝ\left(x,t\right)+g\left(x_{1}\right)u+\text{d}\left(x,t\right),\\ y=x_{1}. \end{array}\right) \end{array}$$

Arranging (6) gives

(16) $$\begin{array}{c} \left\{\begin{array}{c} {\dot{x}}_{1}=x_{2},\\ {\dot{x}}_{2}=F+b_{0}u+b_{0}\text{d,}\\ y=x_{1}. \end{array}\right) \end{array}$$

Let

(17) $$\begin{array}{c} x_{3}=ℱ+b_{0}\text{d}. \end{array}$$

Thus, substituting equations (18) into (16) yields

(18) $$\begin{array}{c} \left\{\begin{array}{c} {\dot{x}}_{1}=x_{2},\\ {\dot{x}}_{2}=x_{3}+b_{0}u,\\ y=x_{1}. \end{array}\right) \end{array}$$

Differentiating (19) thus gives

(19) $$\begin{array}{c} {\dot{x}}_{3}=\dot{ℱ}+b_{0}\dot{\text{d}}, \end{array}$$

(20) $$\begin{array}{c} \left\{\begin{array}{c} {\dot{x}}_{2}=x_{3}+b_{0}u,\\ {\dot{x}}_{3}=\dot{ℱ}+b_{0}\dot{\text{d}}, \end{array}\right) \end{array}$$

where *x*_3_ is the generalized disturbance, ℱ represents the system dynamics and parameter uncertainty, and d is the exogenous disturbance.

The general form of equations (13) and (14) can be rewritten as

(21) $$\begin{array}{c} \left\{\begin{array}{c} {\dot{z}}_{1}=z_{2}+\beta_{1}{\hat{e}}_{1},\\ {\dot{z}}_{2}=z_{3}+\beta_{2}{\hat{e}}_{2},\\ \vdots ,\\ {\dot{z}}_{\rho }=z_{\rho +1}+b_{0}u+\beta_{\rho }{\hat{e}}_{\rho },\\ {\dot{z}}_{\rho +1}=\beta_{\rho +1}{\hat{e}}_{\rho +1}, \end{array}\right) \end{array}$$

where *ρ* is the relative degree of the system, *z*_*ρ*_ is the estimated state of *x*_*ρ*_, and *z*_*ρ*+1_ is the estimated total disturbance. $\text{To achieve this},\;{\hat{e}}_{1,2\cdots \rho +1}$ is a nonlinear function that can be expressed as

(22) $$\begin{array}{c} \left\{\begin{array}{c} {\hat{e}}_{1}=\text{sign}\left(e_{1}\right){\left|e_{1}\right|}^{\rho_{1}}+Ae_{1},\\ {\hat{e}}_{2}=\text{sign}\left(e_{1}\right){\left|e_{1}\right|}^{\rho_{1}/2}+Ae_{1},\\ \vdots \\ {\hat{e}}_{\rho }=\text{sign}\left(e_{1}\right){\left|e_{1}\right|}^{\rho_{1}/\ell }+Ae_{1},\\ {\hat{e}}_{\rho +1}=\text{sign}\left(e_{1}\right){\left|e_{1}\right|}^{\rho_{1}/\ell +1}+Ae_{1}. \end{array}\right) \end{array}$$

The estimated error can thus be written as

(23) $$\begin{array}{c} e_{i}=x_{i}-z_{i}, \end{array}$$

where *i* ∈ {1,2,…, *ρ*+1}, *e*_*i*_ is the estimated error, and *z*_*i*_ is the estimated state of *x*_*i*_, *ℓ* ∈ {1,2,…, *m*}, where *m* is an integer number.

(24) $$\begin{array}{c} \left\{\begin{array}{c} e_{1}=x_{1}-z_{1},\\ e_{2}=x_{2}-z_{2},\\ \vdots \\ e_{\rho }=x_{\rho }-z_{\rho },\\ e_{\rho +1}=x_{\rho +1}-z_{\rho +1}. \end{array}\right) \end{array}$$

Differentiating (24) gives

(25) $$\begin{array}{c} \left\{\begin{array}{c} {\dot{e}}_{1}={\dot{x}}_{1}-{\dot{z}}_{1},\\ {\dot{e}}_{2}={\dot{x}}_{2}-{\dot{z}}_{2},\\ \vdots \\ {\dot{e}}_{\rho }={\dot{x}}_{\rho }-{\dot{z}}_{\rho },\\ {\dot{e}}_{\rho +1}={\dot{x}}_{\rho +1}-{\dot{z}}_{\rho +1}. \end{array}\right) \end{array}$$

ℒ=*x*_3_ can be used to describe the generalized disturbance, and substituting (21) into (25) yields

(26) $$\begin{array}{c} \left\{\begin{array}{c} {\dot{e}}_{1}=x_{2}-z_{2}-\beta_{1}{\hat{e}}_{1},\\ {\dot{e}}_{2}=x_{3}-z_{3}-\beta_{2}{\hat{e}}_{2},\\ \vdots \\ {\dot{e}}_{\rho }=x_{\rho +1}+b_{0}u-z_{\rho +1}-b_{0}u-\beta_{\rho }{\hat{e}}_{\rho },\\ {\dot{e}}_{\rho +1}=\dot{ℒ}-\beta_{\rho +1}{\hat{e}}_{\rho +1}. \end{array}\right) \end{array}$$

Simplifying (26) goes to

(27) $$\begin{array}{c} \left\{\begin{array}{c} {\dot{e}}_{1}=e_{2}-\beta_{1}{\hat{e}}_{1},\\ {\dot{e}}_{2}=e_{3}-\beta_{2}{\hat{e}}_{2},\\ \vdots \\ {\dot{e}}_{\rho }=e_{\rho +1}-\beta_{\rho }{\hat{e}}_{\rho },\\ {\dot{e}}_{\rho +1}=\dot{ℒ}-\beta_{\rho +1}{\hat{e}}_{\rho +1}. \end{array}\right) \end{array}$$

Expressing (27) in matrix form yields

(28) $$\begin{array}{c} \dot{e}={Α}_{0}e+{Α}_{d}\dot{ℒ}. \end{array}$$

Assuming ${\hat{e}}_{1}={Κ}_{1}\left(e_{1}\right),\ldots$, ${\hat{e}}_{\rho }={Κ}_{\rho }\left(e_{1}\right)$ and ${\hat{e}}_{\rho +1}={Κ}_{\rho +1}\left(e_{1}\right)$.

Then

(29) $$\begin{array}{c} {Α}_{0}=\left[\begin{array}{ccccc} -\beta_{1}{Κ}_{1}\left(e_{1}\right) & 1 & \ldots & 0 & 0\\ -\beta_{2}{Κ}_{2}\left(e_{1}\right) & 0 & \ddots & 0 & 0\\ \vdots & \vdots & \; & \vdots & \vdots \\ -\beta_{\rho }{Κ}_{\rho }\left(e_{1}\right) & 0 & \ldots & 0 & 1\\ -\beta_{\rho +1}{Κ}_{\rho +1}\left(e_{1}\right) & 0 & \ldots & 0 & 0 \end{array}\right],\\ {Α}_{d}=\left[\begin{array}{c} 0\\ \begin{array}{c} \vdots \\ \begin{array}{c} 0\\ 1 \end{array} \end{array} \end{array}\right],\\ \dot{e}=\left[\begin{array}{ccc} {\dot{e}}_{1} & \cdots & {\dot{e}}_{\rho +1} \end{array}\right],\\ e=\left[\begin{array}{ccc} e_{1} & \cdots & e_{\rho +1} \end{array}\right]. \end{array}$$

In order to check if the estimated error converges to zero at *t*⟶*∞*, the Lyapunov stability test can be used [29]. Taking the Lyapunov function *V*_NLESO_=1/2*e*^*T*^*e* and ${\dot{V}}_{\text{NLESO}}=e^{T}\dot{e}$.

So that for *ρ*=1

(30) $$\begin{array}{c} {\dot{V}}_{\text{NLESO}}=\left[\begin{array}{cc} e_{1} & e_{2} \end{array}\right]\left[\begin{array}{cc} -\beta_{1}{Κ}_{1}\left(e_{1}\right) & 0\\ -\beta_{2}{Κ}_{2}\left(e_{1}\right) & 1 \end{array}\right]\left[\begin{array}{c} e_{1}\\ e_{2} \end{array}\right]+\dot{ℒ}. \end{array}$$

Assuming that $\dot{ℒ}$ converges to zero as *t*⟶*∞*, which is the case for constant exogenous disturbances, then

(31) $$\begin{array}{c} {\dot{V}}_{\text{NLESO}}=\left[\begin{array}{cc} e_{1} & e_{2} \end{array}\right]\left[\begin{array}{cc} -\beta_{1}{Κ}_{1}\left(e_{1}\right) & 0\\ -\beta_{2}{Κ}_{2}\left(e_{1}\right) & 1 \end{array}\right]\left[\begin{array}{c} e_{1}\\ e_{2} \end{array}\right]. \end{array}$$

The quadric form, ${\dot{V}}_{\text{NLESO}}=e^{T}Q\dot{e}$, is asymptotically stable if *Q* is a negative definite matrix, which causes the system to be asymptotically stable.

To check whether the *Q* matrix is negative definite and to find its stability limits, the Routh stability criteria can be used. It is first necessary to compute the characteristic equation for matrix *Q* as

(32) $$\begin{array}{c} \left|\lambda Ι-Q\right|=0,\\ \left|\begin{array}{cc} \lambda +\beta_{1}{Κ}_{2}\left(e_{1}\right) & -1\\ \beta_{2}{Κ}_{2}\left(e_{1}\right) & \lambda \end{array}\right|=0. \end{array}$$

Analyzing using the Routh stability criteria yields Table 1.

(33) $$\begin{array}{c} \lambda^{2}+\beta_{1}{Κ}_{1}\left(e_{1}\right)\lambda +\beta_{2}{Κ}_{2}\left(e_{1}\right)=0,\\ \beta_{1}{Κ}_{1}\left(e_{1}\right)>0,\beta_{1}>0,\beta_{2}{Κ}_{2}\left(e_{1}\right)>0,\beta_{2}>0, \end{array}$$

where *Q* is thus negative definite if the *β*_1_ and *β*_2_ > 0. Based on this, it can be determined that the NLESO is asymptotically stable.

### 4.2. Closed-Loop Stability Analysis

In this subsection, the closed-loop stability of the overall system is analyzed and proved using the Lyapunov stability criterion.

Taking a nonlinear system as given in equations (1)–(7), where *ρ*=1, the error dynamic of the closed-loop system can be written as

(34) $$\begin{array}{c} \tilde{e}=r-z_{1}. \end{array}$$

Differentiating (34) yields

(35) $$\begin{array}{c} \dot{\tilde{e}}=\dot{r}-{\dot{z}}_{1}. \end{array}$$

Simplifying (35) thus gives

(36) $$\begin{array}{c} \dot{\tilde{e}}=-z_{2}-b_{0}u. \end{array}$$

**Assumption 1 .**

The tracking differentiator in equation (8) tracks the reference error signal with a very small error that approaches zero and with $\dot{\tilde{e}}=0$.

(37) $$\begin{array}{c} \underset{t⟶\infty }{\lim}\left|{\tilde{e}}_{1}-\tilde{e}\right|=0. \end{array}$$

**Assumption 2 .**

The NLESO in equation (12) estimates all states of the nonlinear system.

(38) $$\begin{array}{c} \underset{t⟶\infty }{\lim}e_{1}=0. \end{array}$$

**Theorem 1 .**

Taking the nonlinear system given in equation (14) and the modified ADRC as a basis, then, based on assumptions 1 and 2, the closed-loop system is stable if $\left\{{𝒦}_{1}\left({\tilde{e}}_{1}\right){\tilde{e}}_{1},{𝒦}_{2}\left({\tilde{e}}_{2}\right){\tilde{e}}_{2}\right\}$ is chosen in such a way that the *Q* matrix is negative definite and satisfies the characteristic equation $\lambda^{2}+\lambda \left(\overset{\prime }{{𝒦}_{1}}+\overset{\prime }{{𝒦}_{2}}\right)+\overset{\prime }{{𝒦}_{1}}\overset{\prime }{{𝒦}_{2}}=0$.

**Proof**

Taking *u*=*u*_0_ − *z*_2_/*b*_0_, equation (36) can be rewritten as

(39) $$\begin{array}{c} \dot{\tilde{e}}=-z_{2}-b_{0}\left[u_{0}-\frac{z_{2}}{b_{0}}\right]. \end{array}$$

Simplifying (39) thus gives

(40) $$\begin{array}{c} \dot{\tilde{e}}=-b_{0}u_{0}, \end{array}$$

Eq. (40) when substituting the NLPID in Eq. (10) or STC-SM Eq. (12) is introduced next and stated as follows.

#### 4.2.1. With NLPID-TD

**Remark 1 .**

The extended state of the NLESO *z*_2_ approaches the generalized disturbance ℒ and cancels it in an online manner with a steady-state error, *e*_2_, that converges to zero as *t*⟶*∞*, converting the system in equation (14) into a chain of integrators, thus removing the need for integrator term *u*_3_ in the proposed NLPID controller as seen in equation (9). The NLPD used in this paper is thus expressed as follows:

(41) $$\begin{array}{c} \left\{\begin{array}{c} u_{0_{\text{NLPD}}}=u_{1}+u_{2},\\ u_{1}=\frac{k_{1}}{1+\exp\left({\tilde{e}}_{1}^{2}\right)}{\left|{\tilde{e}}_{1}\right|}^{\alpha_{1}}\text{sign}\left({\tilde{e}}_{1}\right),\\ u_{2}=\frac{k_{2}}{1+\exp\left({\dot{\tilde{e}}}_{1}^{2}\right)}{\left|{\dot{\tilde{e}}}_{1}\right|}^{\alpha_{2}}\text{sign}\left({\dot{\tilde{e}}}_{1}\right). \end{array}\right) \end{array}$$

Substituting (41) into (40) gives

(42) $$\begin{array}{c} \dot{\tilde{e}}=-b_{0}\left[u_{1}\left({\tilde{e}}_{1}\right)+u_{2}\left({\tilde{e}}_{2}\right)\right]. \end{array}$$

**Assumption 3 .**

Assume ${𝒦}_{i}\left({\tilde{e}}_{i}\right)=k_{i}/1+\text{exp}\left({\tilde{e}}_{i}^{2}\right)$, *i* ∈ {1, 2}, with *α*_1_ and *α*_2_ assumed to approach unity: thus, the term |*𝕊*|sign(*𝕊*) in (41) is approximately equal to *𝕊*, allowing equation (42) to be rewritten as

(43) $$\begin{array}{c} \dot{\tilde{e}}=-b_{0}\left[K_{1}\left({\tilde{e}}_{1}\right){\tilde{e}}_{1}+K_{2}\left({\tilde{e}}_{2}\right){\tilde{e}}_{2}\right]. \end{array}$$

Expressing (36) in matrix form gives $\dot{\tilde{e}}=A_{C_{\text{NLPD}}}\tilde{e},$ where $A_{C_{\text{NLPD}}}=\left[\begin{array}{cc} -{𝒦}_{1}^{\prime } & -{𝒦}_{2}^{\prime } \end{array}\right]$ and $\tilde{e}=\left[\begin{array}{c} {\tilde{e}}_{1}\\ {\tilde{e}}_{2} \end{array}\right]$, ${𝒦}_{i}^{\prime }=b_{0}{𝒦}_{i}\left({\tilde{e}}_{i}\right),\;i\in \left\{1,2\right\}$.

The Lyapunov function is then used to check the stability of the closed-loop system:$V_{\text{cl}}=1/2{\tilde{e}}^{T}\tilde{e}$, so that ${\dot{V}}_{\text{cl}}={\tilde{e}}^{T}\dot{\tilde{e}}$.

(44) $$\begin{array}{c} {\dot{V}}_{\text{cl}}=\left[\begin{array}{cc} {\tilde{e}}_{1} & {\tilde{e}}_{2} \end{array}\right]\left[\begin{array}{cc} -K_{1}^{\prime } & -K_{2}^{\prime } \end{array}\right]\left[\begin{array}{c} {\tilde{e}}_{1}\\ {\tilde{e}}_{2} \end{array}\right]. \end{array}$$

The quadric form ${\dot{V}}_{cl}={\tilde{e}}^{T}Q\dot{\tilde{e}}$ is stable if *Q* is a negative semidefinite matrix, causing the whole system to be stable.

To verify the negative definiteness of *Q*, the Routh stability criteria (Table 2) can be used. This requires completing the characteristic equation for matrix *Q* and computing it as follows:

(45) $$\begin{array}{c} \left|\lambda Ι-\text{Q}\right|=0,\\ \left|\begin{array}{cc} \lambda & 0\\ 0 & \lambda \end{array}\right|-\left|\begin{array}{cc} -\overset{\prime }{K_{1}} & 0\\ 0 & -\overset{\prime }{K_{2}} \end{array}\right|,\\ \lambda^{2}+\lambda \left(\overset{\prime }{K_{1}}+\overset{\prime }{K_{2}}\right)+\overset{\prime }{\overset{\prime }{K_{1}}\overset{\prime }{K_{2}}}=0, \end{array}$$

The system is stable if the nonlinear function gains *𝒦*_1_′ and *𝒦*_2_′ satisfy the conditions noted above.

(46) $$\begin{array}{c} \overset{\prime }{K_{1}}\overset{\prime }{K_{2}}>0\Rightarrow_{1}>0\text{or}\\ K_{2}>0. \end{array}$$

#### 4.2.2. With the Proposed STC-SM

STC-SM substitution of equation (11) into equation (40) yields

(47) $$\begin{array}{c} \dot{\tilde{e}}=-b_{0}\left[\kappa {\left|\varsigma \right|}^{\rho }\text{sign}\left(\varsigma \right)+\xi \text{tan}h\left(\frac{\varsigma }{\delta }\right)\right], \end{array}$$

where $\varsigma =\kappa {\tilde{e}}_{1}+{\dot{\tilde{e}}}_{1}$.

As noted previously, the Lyapunov function was used to check the stability of the closed-loop system:

If *V*_cl_=1/2*ς*^*T*^ *ς*, then ${\dot{V}}_{cl}=\varsigma^{T}\dot{\varsigma }$. Given $\dot{\varsigma }=u_{0_{\text{STC}-\text{SM}}}$, Then ${\dot{V}}_{\text{cl}}=\varsigma^{T}\left[-\kappa {\left|\varsigma \right|}^{\rho }\text{sign}\left(\varsigma \right)-\xi \text{tan}h\left(\varsigma /\delta \right)\right]$.

(48) $$\begin{array}{c} {\dot{V}}_{\text{cl}}=-\kappa {\left|\varsigma \right|}^{\rho +1}\text{sign}\left(\varsigma \right)-\varsigma \xi \text{tan}h\left(\frac{\varsigma }{\delta }\right), \end{array}$$

where ${\dot{V}}_{\text{cl}}<0\text{ if }\kappa$ and *ξ* > 0,  and the system is stable.

## 5. Simulation Results and Discussion

The proposed ADRC and proposed COVID-19 nonlinear model were designed and simulated using MATLAB/Simulink. The parameters of the COVID-19 model are shown in Table 3, based on estimated data from Italy [17]. The simulations included comparing the proposed schemes with a nonlinear ADRC. In this paper, the performance of each overall system is measured using the multiobjective performance index (OPI), expressed as follows:

(49) $$\begin{array}{c} \text{OPI}=W_{1}*\frac{\text{IAU}}{N_{1}}+W_{2}*\frac{\text{ISU}}{N_{2}}, \end{array}$$

where *W*_1_ and *W*_2_ are the weighting factors that satisfy *W*_1_+*W*_2_ = 1. Based on this, they are set to *W*_1_ = 0.6 and *W*_2_ = 0.4, while *N*_1_ and *N*_2_ are the nominal values of the individual objective functions, and their values are set to *N*_1_ = 514.250880 and *N*_2_ = 1.449457.  Table 4 shows the description and mathematical representation of all performance indices. The simulation was done with initial value *S*(0)=9,979000, *E*(0)=2,000000, *I*(0)=1000, *R*(0)=0, *H*(0)=0, *C*(0)=0, and *D*(0)=0.

In this paper, three schemes are used, expressed as follows:

(1) Scheme 1: Nonlinear state error feedback (NLADRC) [18] + linear ESO (LESO). The LESO can be expressed as
  (50) $$\begin{array}{c} \left\{\begin{array}{c} {\dot{z}}_{1}=z_{2}+b_{0}u+\beta_{1}\left(e_{1}\right),\\ {\dot{z}}_{2}=\beta_{2}\left(e_{1}\right), \end{array}\right) \end{array}$$
  while the NLSEF of [18] can be expressed as
  (51) $$\begin{array}{c} \left\{\begin{array}{c} \text{fal}\left({\tilde{e}}_{1},\alpha_{1},\delta_{1}\right)=\left\{\begin{array}{cc} \frac{{\tilde{e}}_{1}}{\left(\delta_{1}^{1-\alpha_{1}}\right)}, & x\leq \delta_{1},\\ {\left|{\tilde{e}}_{1}\right|}^{\alpha_{1}}\text{sign}\left({\tilde{e}}_{1}\right), & x>\delta_{1}, \end{array}\right.\\ u_{0}=\text{fal}\left({\tilde{e}}_{1},\alpha_{1},\delta_{1}\right),\\ u_{1}=u_{0_{\text{NLSEF}}}-\frac{z_{2}}{b_{0}}, \end{array}\right. \end{array}$$
  where ${\tilde{e}}_{1}=r-z_{1}$, *e*_*i*2_ is the tracking error, *α*_1_ and *δ*_1_ are positive tuning parameters, and *β*_1_ and *β*_2_ are the observer gain parameters.
(2) Proposed Scheme 1: The NLESO of equations (13) and (14) + NLPD of (41) + TD of (2).
(3) Proposed Scheme 2: The NLESO of equations (13) and (14) + STC-SM of equations (11) and (12) + TD of equation (9).

The simulated results for each scheme are given in Tables 5, 6, and 7, along with the tuned parameters of both controllers and observers for the aforementioned schemes.

The simulation was performed to confirm the effectiveness of the vaccination control strategy with different nonlinear controllers and nonlinear ESO in the proposed model, to verify the robustness of the proposed method. The simulation was done with the initial values mentioned previously and an applied disturbance of −10000. As shown in Figures 5(a)–5(g), the number of recovered individuals after about 35 days reached about 12 million, while infected individuals reached about zero after 18 days. Moreover, the number of hospitalized people and exposed people reached zero after 35 days and 24 days, respectively, while the total deaths did not exceed 0.08 million in total within 100 days. Figures 6(a)–6(g) shows almost the same results except for the total death, which increased by 0.043385% of the proposed scheme 1 total death value, but it did not increase after day 35. As shown in Figure 7(a)to 7(g), the proposed schemes (i.e., Figures 6 and 7) together achieve excellent results as compared to scheme 1, where total deaths within 100 days exceed 0.08 million, an increase of about 0.0456%, and it takes about 40 days to arrive at the desired value. In addition, the numbers of exposed, infected, and hospitalized individuals reach zero after about 35–50 days, highlighting the effectiveness of the vaccinations used. As these vaccinations were discovered and developed only recently, proof of effectiveness is required; currently, there is some fear and various questions about the effectiveness of the vaccine or the side effects that may appear in the future and affect people's health, counterbalanced by the fact that some countries or small cities do not have sufficient capability to buy vaccines. These issues can be considered as disturbances, further supporting the effectiveness of the proposed NLESO.

Figure 8 shows the control signal for the proposed scheme 1, proposed scheme 2, and scheme 1. This shows that vaccination within the first 15 days after an outbreak can reduce or suppress the spread of COVID-19 in a highly efficient manner. Moreover, the number of vaccinated individuals per day for the proposed schemes is higher than in scheme 1, with the number of vaccinated individuals at about 2.5 million and 2 million per day for proposed scheme 1 and proposed scheme 2, respectively, while for scheme 1, the number of vaccinated individuals is only about 1.2 million, which proves the success of the proposed controller with respect to achieving a smooth response and excellent results.  Table 8 shows the simulation results for the performance index and OPI.

Table 8 shows the simulated results of the performance indices for the schemes applied in this paper. As shown, the proposed schemes offer improvements in energy-saving, which for this paper and its focus on COVID-19 systems, represent the capability of the vaccines to be stored at the normal temperature of pharmacy refrigerators, which is about −20°*C*. Based on this, the vaccines will be available in a short time in most countries, as the IAU is reduced by 95.75694% and 90.49362% for proposed scheme 1 and proposed scheme 2, respectively, and the ISU is reduced by 98.3729%% and 99.0166% for proposed scheme 1 and proposed scheme 2, respectively. Finally, the proposed schemes also achieve the best values for OPI, IAU, and ISU.

**Remark 2 .**

Although, all the obtained results are perfect, however, there are some difficulties that we faced in this work and can be summarized as follows:

1. The stability of the COVID-19 mathematical model. This issue has been solved by choosing a suitable value for *b*_COV_ and the suitable design of the proposed controller.
2. Tuning of the controller and observer parameters. This issue is solved by making that all the parameters are tuning parameters that tuned using GA [30, 31] and improved the system using the multi-objective performance index OPI.

## 6. Conclusions

The COVID-19 epidemic has spread rapidly in recent years, and the number of infections and deaths around the world increased rapidly at first. The need for vaccines was thus seen to increase day by day, as part of multiple efforts to reduce the spread of COVID-19 and subsequently eliminate the COVID-19 virus. About a year and a half after the first infections, vaccination was made available around the world. In this paper, NLPD and STC-SM are proposed for application to generate proper vaccination control, together with a proposed nonlinear ESO that eliminates the total disturbance to form an ADRC that can be used to contain the spread of COVID-19. The simulation results show that the proposed schemes are very effective in reducing the spread of COVID-19, assuming that the vaccinated individuals have acquired immunity to the virus sufficient that even if they contact infected people, they will not be further infected. The closed-loop stability and convergence of the NLESO are also demonstrated. A proposed extension to this work would include another country with a large population as a case study [32].

## Figures and Tables

**Figure 1:** Flow diagram of COVID-19.

**Figure 2:** ADRC general form.

**Figure 3:** The proposed relative degree one ADRC.

**Figure 4:** The proposed ADRC with a nonlinear model of the COVID-19 system with relative degree *ρ*=1.

**Figure 5:** Simulation results for scheme 1: (a) susceptible individuals, (b) exposed individuals, (c) infected individuals, (d) hospitalized individuals, (e) cumulative infected, (f) recovered individuals, and (g) cumulative deaths due to SARS-CoV-2.

**Figure 6:** Simulation results for proposed scheme 1: (a) susceptible individuals, (b) exposed individuals, (c) infected individuals, (d) hospitalized individuals, (e) cumulative infected, (f) recovered individuals, and (g) cumulative deaths due to SARS-CoV-2.

**Figure 7:** Simulation results for proposed scheme 2: (a) susceptible individuals, (b) exposed individuals, (c) infected individuals, (d) hospitalized individuals, (e) cumulative infected, (f) recovered individuals, and (g) cumulative deaths due to SARS-CoV-2.

**Figure 8:** Control signal.

**Table 1:** Routh stability analysis for *Q* matrix (NLESO case).

1	*β*_2_ *K*_2_(*e*_1_)
*β*_1_Κ_1_(*e*_1_)	0
$\frac{\beta_{2}{Κ}_{2}\left(e_{1}\right)\beta_{1}{Κ}_{1}\left(e_{1}\right)}{\beta_{1}{Κ}_{1}\left(e_{1}\right)}=\beta_{2}{Κ}_{2}\left(e_{1}\right)$	0

**Table 2:** Routh stability analysis for *Q* matrix (closed-loop analysis case).

$\begin{array}{c} \lambda^{2}\\ \lambda \\ \lambda^{0} \end{array}$	$\begin{array}{c} 1\\ \overset{\prime }{{𝒦}_{1}}+\overset{\prime }{{𝒦}_{2}}\\ \frac{\left(\overset{\prime }{{𝒦}_{1}}+\overset{\prime }{{𝒦}_{2}}\right)\overset{\prime }{{𝒦}_{1}}\overset{\prime }{{𝒦}_{2}}}{\overset{\prime }{{𝒦}_{1}}+\overset{\prime }{{𝒦}_{2}}}=\overset{\prime }{{𝒦}_{1}}\overset{\prime }{{𝒦}_{2}} \end{array}$	$\begin{array}{c} \overset{\prime }{{𝒦}_{1}}\overset{\prime }{{𝒦}_{2}}\\ 0\\ 0 \end{array}$

**Table 3:** Sampled parameters for the COVID-19 system.

Parameters	Value	Descriptions
*λ*_COV_	3.3*∗*10^−5^	The per capita birth rate
*β*_COV_	75*∗*10^−2^	The probability of disease transmission per contact (transmission rate)
*γ*_COV_	2*∗*10^−1^	The recovery rate of infectious individuals
*b*_COV_	5*∗*10^−1^	The diagnosis rate
*α*_COV_	6*∗*10^−3^	The SARS-CoV-2 virus-induced average fatality
*μ*_COV_	3.3*∗*10^−5^	The per capita natural death rate
*ϵ*_COV_	2*∗*10^−1^	The rate of progression from *E* to *I* (the reciprocal of the incubation period)

**Table 4:** Description and mathematical representation of the performance index.

Performance index (PI)	Descriptions	Mathematical representation
IAU	Integral absolute of the control signal	∫_0_^tf^|*u*(*t*)|d*t*
ISU	Integral square of the control signal	∫_0_^tf^*u*(*t*)d*t*

**Table 5:** Scheme 1 parameters.

ADRC part	Parameter	Value
NLSEF	*α*_1_	0.0907
	*δ*_1_	0.7427

LESO	*β*_1_	0.2110
	*β*_2_	0.0111
	*b*_0_	−4.5958

**Table 6:** Proposed scheme 1 parameters.

ADRC part	Parameter	Value	Parameter	Value
NLPD	*k*_1_	6.616000	*k*_2_	4.187500
	*α*_1_	0.084400	*α*_2_	0.339500

TD	*R*	74.7348	*a*_2_	15.5400
	*a*_1_	0.4511	−—	—−

NLESO	*β*_1_	0.97000	*β*_2_	0.235710
	*𝒜*	16.210000	*a*_1_	0.529200
	*b*_0_	−1	—−	—−

**Table 7:** Proposed scheme 2 parameters.

ADRC part	Parameter	Value	Parameter	Value
STC-SM	*κ*	0.164000	*ξ*	1.684000
	*℘*	0.50000	*δ*	6.982000

TD	*R*	5.9990	*a*_2_	0.3280
	*a*_1_	3.1520	—−	—−

NLESO	*β*_1_	6.82000	*β*_2_	12.187081
	*𝒜*	12.140000	*a*_1_	0.423800
	*b*_0_	−8	—−	—−

**Table 8:** Performance indices.

Performance index	Scheme 1	Proposed Scheme 1	Proposed Scheme 2
IAU	15171.563042	641.836188	1442.265125
ISU	230.751769	3.754862	2.269211
OPI	81.380863	1.785072	2.308980

## Data Availability

All data used to support the findings of the study are available within the article.
